This article has been retracted.

# A Femtomol Range FRET Biosensor Reports Exceedingly Low Levels of Cell Surface Furin: Implications for the Processing of Anthrax Protective Antigen

**DOI:** 10.1371/journal.pone.0011305

**Published:** 2010-06-24

**Authors:** Katarzyna Gawlik, Albert G. Remacle, Sergey A. Shiryaev, Vladislav S. Golubkov, Mingxing Ouyang, Yingxiao Wang, Alex Y. Strongin

**Affiliations:** 1 Infectious and Inflammatory Disease Center, Sanford-Burnham Medical Research Institute, La Jolla, California, United States of America; 2 Department of Bioengineering and the Beckman Institute for Advanced Science and Technology, University of Illinois, Urbana-Champaign, Illinois, United States of America; Monash University, Australia

## Abstract

Furin, a specialized endoproteinase, transforms proproteins into biologically active proteins. Furin function is important for normal cells and also in multiple pathologies including malignancy and anthrax. Furin is believed to cycle between the Golgi compartment and the cell surface. Processing of anthrax protective antigen-83 (PA83) by the cells is considered thus far as evidence for the presence of substantial levels of cell-surface furin. To monitor furin, we designed a cleavage-activated FRET biosensor in which the Enhanced Cyan and Yellow Fluorescent Proteins were linked by the peptide sequence SNSRKKR↓STSAGP derived from anthrax PA83. Both because of the sensitivity and selectivity of the anthrax sequence to furin proteolysis and the FRET-based detection, the biosensor recorded the femtomolar levels of furin in the *in vitro* reactions and cell-based assays. Using the biosensor that was cell-impermeable because of its size and also by other relevant methods, we determined that exceedingly low levels, if any, of cell-surface furin are present in the intact cells and in the cells with the enforced furin overexpression. This observation was in a sharp contrast with the existing concepts about the furin presentation on cell surfaces and anthrax disease mechanism. We next demonstrated using cell-based tests that PA83, in fact, was processed by furin in the extracellular milieu and that only then the resulting PA63 bound the anthrax toxin cell-surface receptors. We also determined that the biosensor, but not the conventional peptide substrates, allowed continuous monitoring of furin activity in cancer cell extracts. Our results suggest that there are no physiologically-relevant levels of cell-surface furin and, accordingly, that the mechanisms of anthrax should be re-investigated. In addition, the availability of the biosensor is a foundation for non-invasive monitoring of furin activity in cancer cells. Conceptually, the biosensor we developed may serve as a prototype for other proteinase-activated biosensors.

## Introduction

FRET takes place between a donor and acceptor fluorophore moieties if there is an overlap between the emission spectrum of the donor and the absorption spectrum of the acceptor [1]. In addition to this spectral overlap, the two fluorophores must be properly aligned within a certain distance of each other. There is a close relationship between donor-acceptor distance and efficiency of energy transfer [2], [3], [4]. If the donor and the acceptor are linked by a peptide sequence that spans a proteinase cleavage site, following proteolytic cleavage the donor and the acceptor are separated and are no longer in close proximity. As a result, the level of FRET rapidly and significantly decreases. FRET can be quantified according to a ratio of light emission at the two specific wavelengths which are unique for the donor and the acceptor. These parameters stimulate the use of FRET-based biosensors as the molecular tools in the proteinase research [5], [6], [7], [8], [9], [10], [11], [12].

Multiple cellular proteins including growth factors, hormones, metalloproteinases and cell receptors are synthesized as inactive precursors [13], [14]. These precursors are transformed into functionally active proteins by the cleavage action of proprotein convertases (PCs), specialized serine endoproteinases with the focused cleavage preferences [15], [16]. Seven PCs (furin, PACE4, PC1/3, PC2, PC4, PC5/6, and PC7) have been identified in humans [17]. Furin and other PCs cleave the multibasic motifs Arg-Xxx-Arg/Lys/Xxx-Arg↓, and thus transform proproteins into biologically active proteins and peptides [18], [19], [20], [21]. Furin is currently the most studied enzyme of the PC family. Furin is activated autocatalytically [21]. The autoactivated furin then cleaves latent precursors in the Golgi and the secretory vesicles, and, potentially, also at the cell membrane, post-secretion. In addition to normal cell functions, furin is implicated in many pathogenic states, because it processes to maturity membrane fusion proteins and pro-toxins of a variety of both bacteria and viruses, including anthrax toxin.

Anthrax toxin includes protective antigen and edema and lethal factors (EF and LF, respectively) [22], [23]. It has been suggested that during the process of intoxication, the 83 kDa protective antigen monomer (PA83) binds to the cell surface anthrax toxin receptors. Two receptor types are a capillary morphogenesis protein 2 (CMG2) that is the major receptor mediating lethality of anthrax toxin *in vivo* and the anthrax toxin receptor/tumor endothelial marker 8 (ATR/TEM8) that plays a minor role. CMG2 is expressed in most human tissues. The expression of TEM8 is restricted to tumor endothelium and cancer cells [24]. The receptor-bound PA83 is believed to be then cleaved by cellular furin and related PCs [25], [26]. This cleavage releases a 20 kDa N-terminal fragment and a cell-bound, C-terminal 63 kDa protein (PA63). The latter oligomerizes into a ring-shaped PA heptamer that exposes the binding sites for EF and LF [27], [28]. The functional heptamer, however, may include both PA63 and PA83 [29]. The N-terminal ends of both EF and LF bind to PA63. The respective C-terminal parts of EF and LF exhibit the adenylate cyclase and the metalloproteinase activity, respectively. A complex formed by the PA63 heptamer and either EF or LF or both is internalized into the cell by receptor-mediated, clathrin-dependent, endocytosis [30]. In the acidified lumen of the endosomes, the heptamer forms a channel through which EF and LF are transported from the endosomal compartment into the cytoplasm of the host cell. In the cytoplasm, EF and LF produce their toxic effects.

To analyze the role of furin in the PA83 processing in more detail and to develop a specific biosensor for furin–like PC activity, we have specifically selected the enhanced CFP (ECFP) and YPet (a variant of YFP) pair [6], [31]. According to our experience, the ECFP/YPet FRET pair allows the development of biosensors with the significantly enhanced sensitivity [31]. The ECFP and YPet moieties were linked by a specially selected peptide sequence that was highly sensitive to furin proteolysis [26], [32]. Experimental evidence demonstrated that, as a result, we developed a highly selective and sensitive furin biosensor which, in contrast to the fluorescent peptide substrates, allowed continuous and accurate monitoring of furin activity both on tumor cell surfaces and in tumor cell extracts.

The use of the FRET biosensor in a combination with other analytical methods determined the presence of exceedingly low levels of active furin on the cancer cell surface. In contrast to the previous concept, our results suggest that anthrax PA83 is processed by the furin activity in the extracellular milieu rather than directly on the cell surface. This parameter provides an opportunity for the design of anthrax inhibitors which would inactivate extracellular furin without interfering with normal physiological functions of cellular furin and furin-like PCs.

## Materials and Methods

### Materials

Reagents were purchased from Sigma-Aldrich unless indicated otherwise. The fluorescent substrate pyroglutamic acid-Arg-Thr-Lys-Arg-methyl-coumaryl-7-amide (Pyr-RTKR-AMC) was from Peptides International. The furin inhibitor decanoyl-Arg-Val-Lys-Arg-chloromethylketone (dec-RVKR-cmk) was from Bachem. Aprotinin was purchased from Serological Corporation. Anthrax PA83 was purchased from List Biological Laboratories. Human myelin basic protein (18.5 kDa isoform) was from Biodesign. The pET directional TOPO Expression kit was obtained from Invitrogen. The Fugene HD transfection reagent was from Roche Diagnostics. The murine MON-148 monoclonal antibody against the catalytic domain of furin was from Axxora. A rabbit polyclonal GFP antibody that cross-reacts with ECFP and YPet was from Abcam. The peroxidase-conjugated donkey anti-mouse and anti-rabbit IgGs were from Jackson ImmunoResearch Laboratories. The NS2B-NS3 proteinase from West Nile virus (WNV) was purified as reported earlier [33].

### Cloning and plasmid construction

The ECFP-YPet FRET biosensor (GenBank Accession #EU545473) in the pRSETb vector was initially designed for monitoring the activity of membrane type-1 matrix metalloproteinase [6]. This construct was used as a template for constructing the furin biosensor. The SNSRKKR↓STSAGP sequence of anthrax PA83 was inserted by the PCR mutagenesis in the ECFP-YPet construct using the 5′-AGCAACAGCCGTAAAAAACGTAGTACTAGTGCCGGCCCGATGGTGAGCAAGGGCGAGGAG-3′ and 5′- CGGGCCGGCACTAGTACTACGTTTTTTACGGCTGTTGCTGAGCTCTTTGTACAATTCATT-3′ oligonucleotides as the forward and reverse primers, respectively (the sequence coding for the furin cleavage site is underlined). The amplified sequence was inserted into the pET101/D-TOPO expression vector (Invitrogen) and N-terminally tagged with the Hisx6 and FLAG tags. The authenticity of the constructs was confirmed by DNA sequencing. The constructs encoding the full-length human furin (furWT) and the catalytically inert furin mutant D153N (furD153N) in which Asn replaced the essential active site Asp153 were described earlier [34]. The furin constructs were sub-cloned into the pcDNA 3.1/V5-His-TOPO vector.

### Cells

Human glioma TP98G, U373 and U251, fibrosarcoma HT1080, breast carcinoma MCF-7 and colon carcinoma LoVo cells (all from ATCC, Manassas, VA) were grown in DMEM supplemented with 10% fetal bovine serum (FBS) and penicillin-streptomycin (100 units/ml and 100 µg/ml, respectively). Sub-confluent MCF-7 and LoVo cells (2×10^5^ and 5×10^5^, respectively) were transfected using Fugene HD reagent (3 µl/1 µg DNA). MCF-7 and LoVo cells were transfected with the furWT and furD153N constructs to obtain the stably transfected MCF-7:furWT, MCF-7:furD153N and LoVo:furWT cells. Transfected cells were grown for 3–4 weeks in the presence of G418 (1 mg/ml). Cell clones with the high expression of furin were identified using Western blotting with the furin MON-148 antibody. Glioma U251 cells stably transfected with α1-anti-trypsin variant Portland (a potent inhibitor of furin; PDX) were constructed and characterized earlier (U251/PDX cells) [35], [36].

### Furin biosensor expression and purification

The biosensor construct was expressed in *E. coli* BL21 (DE3) Codon Plus cells. The expression of the construct was induced for 16 h at 30°C using 1 mM isopropyl β-D-thiogalactoside. The cells were collected by centrifugation and disrupted by sonication on ice in 20 mM Tris-HCl buffer, pH 8.0, containing 200 mM NaCl, a proteinase inhibitor cocktail and lysozyme (5 mg/ml). The biosensor was purified from the supernatant fraction using a HiTrap Co^2+^-chelating Sepharose FastFlow 1.6×2.5 cm size column (GE Healthcare) equilibrated with 20 mM Tris-HCl buffer, pH 8.0, containing 200 mM NaCl. The biosensor was eluted using a 25–500 mM gradient of imidazole concentrations in 20 mM Tris-HCl buffer, pH 8.0, containing 200 mM NaCl. The peak fractions were combined, dialyzed against 100 mM Hepes, pH 7.5, containing 150 mM NaCl, 1 mM CaCl_2_, and 1 mM MgCl_2_, and frozen at −80°C until use.

### Furin expression and purification

The expression of the soluble C-terminally truncated furin construct in Sf9 insect cells (an ovarian cell line from fall armyworm *Spodoptera frugiperda*) infected with the recombinant baculovirus and purification of furin were described earlier [34].

### FRET assay

The biosensor (100 pmol; 6 µg) was co-incubated for 15–240 min with purified furin (10–100 fmol; 0.6–6 ng) at 37°C in 0.1 ml of the assay buffer (100 mM Hepes, pH 7.5, containing 150 mM NaCl, 1 mM CaCl_2_ and 1 mM MgCl_2_) in a well of a 96-well plate. The emission ratio of ECFP/YPet (476 nm/526 nm) at λ_ex_ = 437 nm was measured by a fluorescence plate reader (FlexStation3, Molecular Devices) to assess the FRET efficiency between ECFP (serving as a donor) and YPet (serving as an acceptor).

### Cleavage of protein substrates

The cleavage reactions (22 µl each) were performed in 100 mm HEPES, pH 7.5, containing 1 mm CaCl_2_, 1 mm β-mercaptoethanol and 0.005% Brij35 (for furin) and 10 mM Tris-HCl, 8.0 containing 20% glycerol (for WNV NS2B-NS3 proteinase). The ECFP/YPet biosensor and PA83 (20 pmol each) were each co-incubated for 1 h at 37°C with the proteinases at a 1∶1-1∶10,000 enzyme-substrate molar ratio. The cleavage reactions were stopped using 1% SDS. The digests were analyzed by SDS-gel electrophoresis followed by Coomassie staining. Where indicated, aprotinin and dec-RVKR-cmk (at a 1∶4-1∶1,100 and a 1∶20 enzyme-inhibitor molar ratio, respectively) were added to the reactions.

### Cleavage of the biosensor by cell samples

Cells (5×10^4^) in DMEM-10% FBS were seeded in wells of a 96-well plate for 24 h. After washing, 0.1 ml 100 mM Hepes, pH 7.5, supplemented with 150 mM NaCl, 1 mM CaCl_2_, and 1 mM MgCl_2_, 1% insulin-transferrin-selenium liquid supplement (ITS) and the biosensor (100 pmol, 6 µg) were added to the cells. After incubation for 2–16 h, the emission ratio of ECFP/YPet (476 nm/526 nm) at λ_ex_ = 437 nm was measured using a FlexStation3 fluorescence plate reader.

For the cleavage of the biosensor by the cell lysates, the cells were detached using 2% EDTA in PBS. After washing, cells were collected by centrifugation and lysed for 1 h at 4°C in 100 mM Hepes, pH 7.5, supplemented with 150 mM NaCl, 1 mM CaCl_2_, 1 mM MgCl_2_ and 0.1% Triton X-100. The cell lysates (50 µg total protein) were co-incubated for 2 h at 37°C with the biosensor (100 pmol, 6 µg). The emission ratio of ECFP/YPet (476 nm/526 nm) at λ_ex_ = 437 nm was measured using a FlexStation3 fluorescence plate reader. The samples were also analyzed by Western blotting with the anti-GFP antibody.

### Processing of PA83 by the cells

PA83 was labeled for 30 min at 4°C using EZ-Link sulfo-NHS-LC-biotin (Pierce; a 1∶20 protein-biotin molar ratio). Excess biotin was removed using a 0.7-ml spin-column. Where indicated, biotin-labeled PA83 (bPA83) was co-incubated with furin (at a 1∶100 enzyme-substrate molar ratio) to convert bPA83 into biotin-labeled PA63 (bPA63). U251, LoVo-mock and LoVo:furWT cells (3×10^5^) were each incubated for 3 h at 37°C in DMEM supplemented with 25 mM HEPES, pH 7.0, 0.2% BSA and bPA63 or bPA83 (1 µg/ml). Where indicated, dec-RVKR-cmk (25 µM) and aprotinin (100 µM) were added to the cells 20 min before adding bPA83/bPA63. After incubation, cells were lysed in 50 mM octyl-β-D-glucopyranoside (Amresco) in TBS supplemented with 1 mM CaCl_2_, 1 mM MgCl_2_, a protease inhibitor mixture set III, 1 mM phenylmethylsulfonyl fluoride (PMSF) and dec-RVKR-cmk (5 µM). To measure cell-associated bPA83 and bPA63, the samples were analyzed by Western blotting with horseradish peroxidase-conjugated ExtrAvidin and a TMB/M substrate (Chemicon). Where indicated, cells were washed for 3 min in 50 mM glycine-100 mM NaCl, pH 3.0, to remove cell surface-associated bPA83/bPA63. The samples were then neutralized using 500 mM Hepes-100 mM NaCl, pH 7.5 [37].

### Cell surface biotinylation

Cells (15×10^6^; 90% confluent) were washed twice with an ice-cold Soerensen Buffer (SBS), pH 7.8, containing 14.7 mm KH_2_PO_4_, 2 mm Na_2_HPO_4_, and 120 mm sorbitol, and then incubated for 10 min in ice-cold SBS. Cell surface-associated furin was biotinylated by incubating cells for 25 min on ice with SBS supplemented with membrane-impermeable EZ-Link NHS-LC-biotin (0.3 mg/ml). Excess biotin was removed by washing the cells in SBS. The residual amounts of biotin were quenched by incubating the cells for 10 min in SBS-100 mm glycine. Quenched cells were lysed in 50 mm *N*-octyl-β-d-glucopyranoside in 50 mM Tris-HCl, pH 7.4, supplemented with 150 mM NaCl, 1 mm CaCl_2_, 1 mm MgCl_2_, a proteinase inhibitor cocktail set III, 1 mm PMSF and 10 µM dec-RVKR-cmk. Biotin-labeled furin was precipitated from the cell lysates using streptavidin-agarose beads. The precipitated samples were analyzed by Western blotting with the MON-148 furin antibody followed by donkey anti-mouse IgG-conjugated with horseradish peroxidase and a SuperSignal West Dura Extended Duration Substrate kit (Pierce).

### Peptide substrate cleavage

The cleavage reactions (200 µl each) were performed in 100 mm HEPES, pH 7.5, containing 1 mm CaCl_2_, 1 mm β-mercaptoethanol and 0.005% Brij-35 (for furin) and 10 mM Tris-HCl, 8.0 containing 20% glycerol (for WNV NS2B-NS3 proteinase). Pyr-RTKR-AMC (25 µM) was used as a substrate. The assays were performed in triplicate in wells of a 96-well plate. The steady-state rate of substrate hydrolysis was monitored continuously at λ_ex_ = 360 nm and λ_em_ = 465 nm at 37°C using a fluorescence plate reader.

### Cell viability assay

Cells (5×10^4^) were grown in DMEM-10% FBS for 16 h in wells of a 96-well plate. After washing, the cells were incubated for 2–4 h in 100 mM Hepes, pH 7.5, supplemented with 150 mM NaCl, 1 mM CaCl_2_, 1 mM MgCl_2_ and 1% ITS. Cell viability was determined using an ATP-Lite kit (Perkin-Elmer). The resulting luminescence was measured using a plate reader (SpectroFluor Plus, Tecan). Each datum point represented the results of at least three independent experiments performed in triplicate.

### Antibody uptake and immunofluorescence microscopy

Cells were seeded on 13 mm round glass coverslips and grown at 37°C until a 50% confluence. Cells were then washed in PBS, fixed with 4% paraformaldehyde for 15 min, and permeabilized for 4 min using 0.1% Triton X-100. Cells were blocked with 3% BSA and incubated for 16 h at 4°C with the primary antibodies (dilution 1∶1,000-1∶1,500) followed by an 1 h incubation with the secondary species–specific IgG conjugated with Alexa Fluor 488 or Alexa Fluor 594 (Molecular Probes). The slides were mounted in the VectaShield anti-fading embedding medium (Vector Laboratories) containing 4′,6-diamidino-2-phenylindole (DAPI) for the nuclear staining.

In the antibody uptake experiments, cells were incubated for 15 min at 4°C in the serum-free, L-15 medium supplemented with 1% ITS. Cells were next incubated for an additional 1 h at 4°C with the MON-148 furin antibody (10 µg/ml). After washing with ice-cold PBS, the cells were next transferred to 37°C for 1 h to stimulate the antibody uptake. Following fixation and permeabilization as above, the cells were stained for 1 h using the Alexa Fluor 594-conjugated secondary antibody, mounted in the VectaShield medium. Images were acquired using a ×400 original magnification on an Olympus BX51 fluorescence microscope equipped with an Olympus MagnaFire digital camera and MagnaFire 2.1C software.

## Results

### Biosensor design, expression and purification

According the observation by us and others, anthrax PA83 is one of the most sensitive cleavage targets of furin and related PCs [26], [32], [38], [39]. Because the substrate cleavage preferences overlap significantly between furin and other PCs, we refer to furin for simplicity in the text below.

The cleavage of PA83 and its conversion into the N-terminal PA20 and the C-terminal PA63 fragment is a result of the cleavage of the SNSRKKR↓STSAGP sequence by furin [21]. To design an ECFP-YPet biosensor which would be both sensitive to the cleavage by furin and suitable for the FRET-based monitoring of its activity, the C-terminus of YPet and the N-terminus of ECFP were linked by the SNSRKKR↓STSAGP sequence of PA83. To facilitate the isolation of the ECFP-YPet biosensor from the recombinant cells, the construct was N-terminally tagged with the FLAG and Hisx6 tags and expressed in *E.coli*. After induction with isopropyl β-D-thiogalactoside, the biosensor was produced as a soluble protein. After disruption of *E.coli* cells by sonication, the soluble protein fraction was loaded onto a Co^2+^-agarose affinity column. The biosensor protein was eluted with a gradient of imidazole concentrations (Fig. 1).

**Figure 1:** The biosensor and its purification. *Left panel*, the ECFP/YPet construct was N-terminally tagged with the Hisx6 and FLAG tags. The furin cleavage sequence (SNSRKKR↓STSAGP) of anthrax PA83 was inserted between the N-terminal Met of ECFP and the C-terminal Leu of YPet. *Right panel*, SDS-gel electrophoresis of the elution fractions of the biosensor purified by Co^2+^-chelating chromatography.

### The biosensor is cleaved by furin

It is expected that furin would cleave the SNSRKKR↓STSAGP linker sequence and separate YPet and ECFP. These events will decrease FRET and, concomitantly, increase the emission ratio of ECFP/YPet. In agreement, following co-incubation of the biosensor with furin, a decrease in both FRET and the YPet emission was recorded. These events were concomitant with an increase in the ECFP emission. Both the concentration-dependent and time-course studies were consistent with the ratiometric and directly proportional response of the biosensor to furin proteolysis. The levels of furin as low as 10 fmol were sufficient to cause the measurable changes in the ECFP/YPet ratio (Fig. 2).

**Figure 2:** Characterization of the biosensor. *Left panel*, the emission spectra (λ_ex_ = 437 nm) of the purified biosensor (100 pmol) before and after its cleavage for 1 h at 37°C using purified furin (10 fmol and 100 fmol). RFU, relative fluorescence unit. *Middle panel*, the time course of the ECFP/YPet emission ratio (476 nm/526 nm at λ_ex_ = 437 nm) of the biosensor (100 pmol) incubated for 4 h at 37°C with or without furin (10 fmol and 100 fmol). *Right panel*, a ratiometric response of the normalized ECFP/YPet emission ratio to the increasing concentrations of furin. Incubation time, 1 h. These experiments were repeated multiple times with similar results. The representative experiments are shown.

We determined that the biosensor and PA83 were similarly sensitive to furin proteolysis (Fig. 3). There were no cleavage sites in the biosensor additional to the linker and, as a result, only the cleavage products that corresponded to the ECFP and YPet moieties were observed in the digest reactions. Similar to PA83, the biosensor was sensitive to the *in vitro* proteolysis by PACE4, PC1/3, PC2, PC4, PC5/6 and PC7 (data not shown). In turn, both PA83 and the biosensor were resistant to the proteolysis by WNV NS2B-NS3 proteinase regardless that the latter exhibits the furin-like, albeit less stringent, cleavage preferences [33], [40], [41]. In contrast, NS2B-NS3 proteinase and furin were similarly efficient in the cleavage of the fluorescent Pyr-RTKR-AMC peptide substrate (Fig. 4). From these perspectives, the biosensor appeared to be selective for furin and furin-like PCs.

**Figure 3:** The biosensor is cleaved by furin but it is resistant to WNV NS2B-NS3 proteinase. *Left panels*, the biosensor and PA83 were cleaved by furin (1 h; 37°C) at the indicated enzyme-substrate ratio. *Right panel*, the biosensor was cleaved by WNV NS2B-NS3 proteinase (1 h; 37°C) at the indicated enzyme-substrate ratio. The cleavage reactions were analyzed by SDS-gel electrophoresis followed by Coomassie staining.

**Figure 4:** The similar activity of furin and WNV NS2B-NS3 proteinase against Pyr-RTKR-AMC. Both furin and WNV NS2B-NS3 proteinase (0.2-4 pmol each) were allowed to cleave the fluorescent peptide for the indicated time. RFU, relative fluorescence unit.

### The biosensor is activated by cellular furin

Because of its significant, 500-residue, size, the biosensor is incapable of penetrating the plasma membrane efficiently. As a result, we initially used the biosensor to assess cell surface-associated furin in fibrosarcoma HT1080, breast carcinoma MCF-7, and glioma TP98G, U373 and U251 cells, which naturally express different levels of furin and also in colon carcinoma LoVo cells. Because of the two frame-shift mutations in the furin gene, LoVo cells do not express functionally active furin [42]. We also used MCF-7 cells which were stably transfected with either the wild-type furin (MCF-7:furWT) or the catalytically inert furin mutant (MCF-7:furD153N) and LoVo cells with the reconstituted expression of the wild-type furin (LoVo:furWT).

The activity of cellular furin was readily recorded by using the biosensor. A short, 2-h incubation was sufficient for recording furin activity in MCF-7:furWT cells while 8–16 h were required in the cells which express furin naturally. Because of the expression of the catalytically inert furin, both MCF-7:furD153N and LoVo cells did not activate the biosensor. The naturally expressed furin activity was the most prominent in U251 and HT1080 cells (Fig. 5).

**Figure 5:** Activation of the biosensor by cellular furin. Adherent glioma TP98G, U373 and U251 cells, fibrosarcoma HT1080 cells, colon carcinoma LoVo cells and breast carcinoma MCF-7, MCF-7:furD153N and MCF-7:furWT cells (5×10^4^) were co-incubated for 2–16 h with the biosensor (100 pmol).

Based on the ratiometric response curve that shows the normalized ECFP/YPet emission ratio of the biosensor co-incubated for 1 h with the increasing concentrations of purified furin (20–100 fmol) (Fig. 2) and on the data of Fig. 6 that show the normalized ECFP/YPet emission ratio of the biosensor co-incubated for 0.5–4 h with 5×10^4^ MCF-7:furWT cells, it is possible to estimate the number of active furin molecules per cell. Thus, the net activity of furin in 5×10^4^ MCF-7:furWT cells roughly corresponded to 10 fmol (∼0.6 ng) furin or ∼100,000 furin molecules/cell. The level of furin in U251 cells was several-fold lower (Fig. 5). The electrophoretic analysis confirmed the specific cleavage of the biosensor by MCF-7:furWT and U251 cells. The predominant cleavage products correlated with the expected ECFP and YPet moieties (Fig. 6).

**Figure 6:** Activation and cleavage of the biosensor by cellular furin. *Left panel*, the time course of the biosensor cleavage by U251, MCF-7:furWT and MCF-7:fur:D153N cells (5×10^4^). *Right panel*, SDS-gel electrophoresis of the cleavage reactions. Cells (5×10^4^) were incubated for 4 h with the biosensor (100 pmol). After centrifugation, the supernatant samples were separated by SDS-gel electrophoresis followed by Coomassie staining. Purified furin (10 fmol and 100 fmol) was used as a control.

### Low levels of cell surface furin

Western blotting analysis demonstrated that it was difficult to unambiguously detect furin in cell lysates unless the cells with the enforced expression of furin were used (Fig. 7). To determine the levels of cell surface-associated furin, cells were surface-biotinylated using membrane-impermeable biotin. Biotin-labeled proteins were precipitated using the streptavidin-agarose beads. The resulting samples were analyzed by Western blotting with the MON-148 furin antibody. Surprisingly, despite high amounts of the loaded protein material, which corresponded to 12×10^6^cells/lane, exceedingly low levels of furin were detected in the biotin-labeled MCF-7:furWT cell samples (Fig. 7).

**Figure 7:** Analysis of cellular furin. *Left panel*, Western blotting of total cell furin (15 µg total protein that corresponded to 5-7×10^4^ cells depending on a cell type). *Right panel*, Western blotting of cell surface-associated furin. MCF-7 and MCF-7:furWT cells (15×10^6^) were cell surface biotinylated using membrane-impermeable biotin. Biotin-labeled furin was immunoprecipitated from the total cell lysate (TCL) using streptavidin-agarose beads. The beads were washed in 50 mM Tris-HCl, pH 7.4, supplemented with 50 mm *N*-octyl-β-d-glucopyranoside, 150 mM NaCl, 1 mm CaCl_2_, 1 mm MgCl_2_, a proteinase inhibitor cocktail set III, and 1 mm PMSF (FT, flow through fraction). The immunocaptured proteins (IP, immunoprecipitated protein fraction) were eluted using 1% SDS. The fractions were analyzed by Western blotting with the furin MON-148 antibody followed by donkey anti-mouse IgG-conjugated with horseradish peroxidase and a SuperSignal West Dura Extended Duration Substrate kit. The gels were overexposed to demonstrate the presence of cell-surface furin. Right lane, purified furin (1 ng). WB, Western blotting.

To corroborate these data, we next used the furin antibody uptake. For these purposes, U251 cells and MCF-7:furWT, which express low and high level of furin, respectively, were allowed to bind the MON-148 antibody for 1 h at 4°C. After washings to remove the unbound antibody, the cells were moved to 37°C to stimulate the internalization of the cell surface-associated furin-antibody complex. The cells were next fixed, permeabilized and stained with a secondary antibody to determine the sub-cellular localization of the furin-antibody complex. We, however, did not detect any significant immunoreactivity, thus, suggesting that there was no detectable level of furin on the cell surface (Fig. 8A).

**Figure 8:** Furin is expressed in the trans-Golgi network in MCF-7:furWT cells. **A**, *left panels*, the uptake of the MON-148 furin antibody did not reveal cell surface furin in U251 and MCF-7:furWT cells. Cells were allowed to bind the antibody at 4°C. Cells were then incubated at 37°C to stimulate the antibody uptake, fixed, permeabilized and stained with the Alexa Fluor 594-conjugated secondary antibody (red). *Right panels*, staining of cellular furin. Cells were fixed, permeabilized and stained using the MON-148 antibody followed by the Alexa Fluor 594-conjugated secondary antibody. **B**, MCF-7:furWT and MCF-7 cells were fixed, permeabilized and stained using the rabbit polyclonal TGN46 antibody (green) and the MON-148 furin antibody (red). The merged panels show the level of co-localization of furin with TGN46 (a trans-Golgi network marker). Original magnification ×400; the bar, 10 µm. The nuclei were stained with DAPI (blue).

We next use direct immunostaining of the permeabilized MCF-7:furWT and MCF-7 (control) cells with the MON-148 antibody. The presence of the intracellular furin was readily recorded in MCF-7:furWT cells. Co-staining of MCF-7:furWT cells using the MON-148 furin antibody and the TGN46 antibody (a trans-Golgi network marker) demonstrated the presence of furin in the trans-Golgi network and in the intracellular vesicles in the permeabilized cells (Fig. 8B). The staining of MCF-7 cells was clearly negative. Non-permeabilized cells also did not show any furin immunoreactivity in the intracellular compartment and at the cell surface (not shown). Overall, the significant levels of cell surface-furin we detected using the biosensor did not correlate with the results of our other studies.

### Proteinases distinct from furin do not cleave PA83

Based on our data, we tested if cellular serine proteinases with PC-like specificity, but distinct from PCs, contributed to the cleavage of both PA83. To exclude this possibility, we used aprotinin, a potent inhibitor of trypsin-like proteinases, in the i*n vitro* and cell-based cleavage tests. Even exceedingly high levels (at a 1∶1000 enzyme-inhibitor molar ratio) of aprotinin did not affect the PA83-converting activity of furin in the cleavage reactions *in vitro*. In contrast, furin activity was fully repressed by its specific inhibitor, dec-RVKR-cmk (k_i_ = 1 nM), at a low, 1∶20, enzyme-inhibitor molar ratio. Consistent with its inhibitory specificity, aprotinin (a nanomolar range inhibitor of WNV NS2B-NS3 proteinase; k_i_ = 26 nM) [33], [43] blocked this proteinase activity at a low, 1∶20, enzyme-inhibitor molar ratio. Because PA83 is resistant to the viral proteinase, the activity of the latter was determined using myelin basic protein as a substrate (Fig. 9) [33].

**Figure 9:** Aprotinin inhibits WNV NS2B-NS3 proteinase activity but not furin. PA83 (1 µM) and myelin basic protein (MBP; 11 µM) were incubated for 1 h at 37°C with furin (1–10 nM; 1∶100-1∶1,000 enzyme-substrate molar ratio) and WNV NS2B-NS3 proteinase (1.25 µM; 1∶10 enzyme-substrate molar ratio) in the presence of the indicated enzyme-inhibitor molar ratio.

We next examined if aprotinin and dec-RVKR-cmk affected the proteolytic processing of PA83 in U251 and LoVo:furWT cells. For this purposes, bPA83 was co-incubated with either the intact cells or with the cells co-incubated with aprotinin or dec-RVKR-cmk. The amounts of cell-associated bPA83 and bPA63 were determined by Western blotting. The results showed intact U251 and LoVo:furWT cells readily processed the external bPA83. Because of the binding to the anthrax toxin receptor, bPA63 and the residual amounts of intact bPA83 were detected in cell extracts. Dec-RVKR-cmk (25 µM) caused a near complete inhibition of bPA83 in U251 cells. In turn, aprotinin (100 µM) did not show any effect (Fig. 10A). As a result, we concluded that cell surface-associated proteinases distinct from furin-like PCs, did not significantly contribute to the processing of PA83. Because cell-surface levels of furin are exceedingly low (Fig. 7 and 8), these data also suggest that PA83 is cleaved by furin in the extracellular milieu but not on the cell surface, and that the resulting PA63 would be capable of binding with the cells. Thus, our earlier data directly indicate that the levels of furin in fibrosarcoma HT1080 and glioma U251 cells are sufficient to sustain efficient anthrax toxin intoxication [44].

**Figure 10:** Specific processing of PA83 by cellular furin. **A**, LoVo:furWT and U251 cells were co-incubated for 3 h at 37°C with bPA83 (1 µg/ml). Where indicated, cells were pre-incubated for 20 min with dec-RVKR-cmk (25 µM) or aprotinin (100 µM) prior to the addition of bPA83. Cell lysates were examined using Western blotting with horseradish peroxidase-conjugated ExtrAvidin and a TMB/M substrate. **B**, *left panel*, U251 cells were incubated for 3 h at 37°C with bPA83 (1 µg/ml) with or without dec-RVKR-cmk (25 µM). Where indicated, cells were exposed to the acid pH treatment to remove the cell surface-associated bPA83 and bPA63. *Right panel*, conversion of bPA83 into bPA63 using purified furin. The gels were stained with Coomassie. WB, Western blotting. NS, non-specific band.

### Both PA83 and PA63 bind the anthrax toxin receptor

To test this suggestion, U251 cells were allowed to bind the equal amounts of bPA83 and of the pre-made bPA63. To generate bPA63, bPA83 was fully processed in the *in vitro* cleavage reactions using the purified furin (Fig. 10B). The levels of the uptake of bPA83 and bPA63 by the cells were determined using Western blotting of the cell lysates. bPA83 and bPA63 were equally efficiently internalized by the cells. Dec-RVKR-cmk inhibited the processing and uptake of bPA83 by the cells. The inhibitor did not affect the processing and uptake of bPA63. Acid treatment of the cells demonstrated the efficient removal of the cell surface-bound bPA83 while there was no similar effect with bPA63 (Fig. 10B). Taken together, these results indicated that bPA83 was not processed at the cell surface in our cell system. Conversely, these results suggested that bPA83 was processed in the extracellular milieu and that only then the generated bPA63 associated with the anthrax toxin receptor in the cells. These parameters suggested the intracellular furin pool but not the cell surface-associated furin contributed to the measurements in our biosensor cleavage tests.

### Intracellular furin pool interfered with the biosensor cleavage

To test if our suggestion was correct, we incubated the biosensor with the adherent MCF-7:furWT and U251 cells. We then determined the normalized ECFP/YPet emission ratio in the supernatant samples (Fig. 11A). In addition, we incubated the cells alone in the assay buffer. We then tested if the supernatant fraction that contained the released cellular proteins was capable of cleaving the biosensor. These tests suggested that the efficiency of the biosensor cleavage by the adherent cells and by the soluble proteins released by the cells was very similar. It appeared that there was a significant release of intracellular furin and, potentially, additional PCs by the cells because the cells did not survive well under our experimental conditions. In agreement, we detected a significant level of apoptosis in the cells. Cell viability tests revealed that 30–35% cells became apoptotic in the course of a short, 4-h, incubation time and that the cell realizate rather than cell surface-associated furin alone contributed to the biosensor cleavage (Fig. 11B). On the other hand, these results also suggested that the cell-impermeable biosensor can be efficiently used to quantify the total cell furin in the cell lysate samples rather than cell surface-associated furin alone using the intact cells.

**Figure 11:** Furin activity was released by the cells. **A**, the time course of the biosensor cleavage by cell realizate and by adherent MCF-7:furWT and U251 cells. Cells (5×10^4^) were incubated for 2 h in 100 mM Hepes, pH 7.5, containing 150 mM NaCl, 1 mM CaCl_2_, 1 mM MgCl_2_ and 1% ITS. The cells were then separated by centrifugation and the supernatant (realizate) was co-incubated with the biosensor for 0–120 min. Alternatively, adherent cells (5×10^4^) were directly co-incubated with the biosensor. **B**, ATP-Lite cell viability assay. Prior to the assay, MCF-7, MCF-7:furWT and U251 cells were incubated for 2–4 h at 37°C in 100 mM Hepes, pH 7.5, containing 150 mM NaCl, 1 mM CaCl_2_, 1 mM MgCl_2_ and 1% ITS. The level of induced apoptosis was then determined using an ATP-Lite kit.

### The biosensor quantifies total cellular furin in cancer cell lysates

Normally, detergents, including Triton X-100, are required for disrupting the cell membrane and for cell protein solubilization. First, we confirmed that the presence of 0.1% Triton in the reactions did not affect the efficiency of the biosensor cleavage by purified furin as determined by both the measurement of the ECFP/YPet ratio and the SDS-gel electrophoresis of the digest samples and (Fig. 12).

**Figure 12:** The biosensor cleavage in cell lysates. *Left panel*, Triton X-100 (0.1%) does not affect the efficiency of furin proteolysis of the biosensor. The biosensor was co-incubated with purified furin (5 fmol and 50 fmol) for 0-120 min with or without 0.1% Triton X-100. *Right panel*, the biosensor was co-incubated 1 h with purified furin at the indicated enzyme-substrate molar ratio. The digests were analyzed by SDS-gel electrophoresis followed by Coomassie staining. Where indicated, reactions contained 0.1% Triton X-100.

We then prepared the total lysates of MCF-7, MCF-7:furWT, MCF-7:furD153N, LoVo, LoVo:furWT, U251 and U251/PDX cells using 0.1% Triton X-100. Following centrifugation to remove the insoluble material, the supernatant aliquots were directly used to cleave the biosensor. Dec-RVKR-cmk was used to inhibit furin in the cleavage reactions. The lysates of MCF-7, MCF-7:furD153N, LoVo and U251/PDX cells did not cleave the biosensor. In contrast, the biosensor cleavage was readily recorded in MCF-7:furWT, LoVo:furWT and U251 cells. Dec-RVKR-cmk fully suppressed the cleavage of the biosensor in these cells (Fig. 13). According to the calibration curve with purified furin (Fig. 2) and the cleavage data using cell lysates, the net levels of furin were 109 fmol, 43 fmol and 24 fmol in MCF-7:furWT, LoVo:furWT and U251 cells, respectively. It is, however, probable that other PCs also contributed to the biosensor cleavage, especially in U251 cells.

**Figure 13:** The biosensor allows to measure reliably furin activity in cell lysates. The time course of the biosensor cleavage by the MCF-7, LoVo and U251 total cell lysates. The cells were lysed for 1 h at 4°C in the buffer containing 0.1% Triton X-100. The insoluble material was discarded by centrifugation. The supernatant aliquots (50 µg total protein; an equivalent of ∼5×10^4^ cells) were co-incubated for 2 h at 37°C with the biosensor (100 pmol).

In contrast with the biosensor, the fluorescent Pyr-RTKR-AMC peptide substrate cannot be employed with the crude cell samples. Indeed, when Pyr-RTKR-AMC was used, the lysates of U251 and U251/PDX cells were similarly efficient in cleaving Pyr-RTKR-AMC despite the drastically different levels of their furin activity. Similarly, there was no significant difference between of the MCF-7, MCF-7:furWT and MCF-7:furD153N samples if Pyr-RTKR-AMC was used (Fig. 14A).

**Figure 14:** The fluorescent peptide substrate does not allow to measure reliably furin activity in cell lysates. **A**, the cleavage of Pyr-RTKR-AMC by the supernatant aliquots (50 µg total protein for MCF-7 and LoVo cells and 5 µg total protein for U251 cells). RFU, relative fluorescence unit. **B**, the biosensor (100 pmol) was co-incubated for 2 h with the total cell lysates or with the purified furin (100 fmol). The digests were analyzed by Western blotting with the GFP antibody. Where indicated, dec-RVKR-cmk was added to the reactions. WB, Western blotting.

To confirm further that other cellular proteinases which are distinct from PCs did not significantly contribute to the biosensor cleavage, the latter was co-incubated with the totals cell lysates of MCF-7:furWT, LoVo:furWT and U251 cells. The digest samples were then analyzed using Western blotting with a GFP antibody (Fig. 14B). The data confirmed the specific cleavage of the biosensor by the MCF-7:furWT, LoVo:furWT and U231 samples. Dec-RVKR-cmk fully repressed the cleavage. Other cell types did not cleave the biosensor efficiently suggesting that cellular proteinases distinct from furin-like PCs did not contribute significantly to the biosensor cleavage.

## Discussion

Multiple physiologically-relevant proteins are synthesized as latent precursors [14], [45]. These precursors are transformed into active proteins by the cleavage action of furin and related PCs [16]. Furin is also implicated in the processing of many pathogens including anthrax [16], [21], [26], [38], [39]. Furin itself is self-activated [21], and upon activation it cleaves *de novo* synthesized latent precursors in the Golgi compartment and in the secretory vesicles. It was believed that some proportion of the furin molecules cycles between the trans-Golgi compartment and the cell surface, albeit the presence of cell-surface furin was never convincingly demonstrated [46]. Because of the overlapping substrate preferences, there is a redundancy in the PC functionality, albeit distinctive functions of furin have also been reported [47].

Evidence suggests that in multiple cancer types furin overexpression causes an imbalance in the activation of invasion- and proliferation-related cellular substrates leading to acquisition of an advanced malignant phenotype [48], [49], [50], [51], [52]. The multiple effects of furin on cell function have led to a concept that in the course of tumor development and progression furin acts as “a master switch” of the tumorigenic protein functionality. If this concept is valid, furin then could be identified as an important therapeutic target in a number of cancer types. The sensitive and selective read-out technology to reliably monitor furin activity in cells and tissues, however, is not currently available. The absence of a reliable read-out does not allow correlating furin activity with disease progression. It also remains unclear how the activity of furin is coordinated in space and time in the cell compartment.

To shed more light on the furin functionality, we designed and tested a cleavage-activated biosensor to monitor the net activity of furin. The biosensor represents a chimeric protein in which an ECFP and YPet FRET pair is linked by a peptide linker sequence derived from anthrax PA83. We specifically selected this sequence as a linker because the SNSRKKR↓STSAGP furin cleavage site of PA83 is supremely sensitive and selective to the proteolysis by furin and related PCs with the redundant cleavage preferences [26], [32].

The use of the biosensor in a combination with other methodologies have allowed us to determine that the levels of cell surface-associated furin are exceedingly low and that they represent a diminutive fraction of the total cell furin. The detected minuscule cell-surface furin levels are grossly insufficient to accomplish the cell-surface processing of anthrax PA83. Our data directly suggest that, at least in the cell-based systems, PA83 is processed by furin extracellularly. This processing is followed by the binding of the resulting PA63 heptamer or the mixed heptamer that includes both the PA63 and the PA83 subunits to the anthrax receptors [22], [24], [29]. Our data shift a long-term paradigm in the furin biology and anthrax infection [53]. In addition, these novel results provide an opportunity for a design of the specific cell-impermeable furin inhibitors of anthrax. These inhibitors would not interfere with normal cellular function of furin and related PCs in the trans-Golgi compartment [39].

It is now tempting to hypothesize that the release of the intracellular furin pool and, probably, other PCs from the already infected, dying cells is cleverly used by anthrax to support the further avalanche-like propagation of infection. The use of the released PCs instead of cell-surface furin eliminates the spatial constraints that limit the interactions between the membrane-tethered PA83-anthrax receptor complexes and furin at the cell surface.

Our tests demonstrated that the biosensor we designed allowed us to selectively record the cleavage activity using as low as the femtomol levels of furin. This high level of selectivity and sensitivity of the biosensor allowed us to detect furin in the tumor cell lysate samples using as low as thousands of cells, a task that is not possible to accomplish reliably with conventional fluorescent peptide substrates. Because serine proteinases distinct from PCs destroy the biosensor rather than specifically cleave the linker sequence, they do not significantly interfere with the specific action by PCs. The availability of the highly sensitive and selective furin biosensor provides a foundation for the rapid, non-invasive procedures to monitor furin and related proteinases in cancer cells and tumor biopsies. Because furin activity is also important for multiple infectious diseases caused by bacterial and viral pathogens, we suggest that the furin biosensor is applicable for monitoring the activity of furin in a wide range of cells and tissues and in a variety of disease conditions rather than in cancer alone.
